RETRACTED

# The value of Monte Carlo model-based variance reduction technology in the pricing of financial derivatives

**DOI:** 10.1371/journal.pone.0229737

**Published:** 2020-02-27

**Authors:** Yunyu Zhang

**Affiliations:** School of Law, Xiamen University, Xiamen, China; University College London, UNITED KINGDOM

## Abstract

The purpose of the study is to reduce the error in the pricing process of financial derivatives, as well as to obtain more accurate product values, thereby reducing transaction costs, accelerating transaction speed, establishing a larger investment scale, and enabling investors to obtain excellent returns under market conditions as much as possible. Based on the variance reduction technology, a Monte Carlo model that can effectively analyze financial prices is added to analyze price fluctuations and find the optimal holding time for users of financial derivatives, thereby reducing the risk of holding the financial derivatives. The results show that the Monte Carlo model-based variance reduction technology can significantly improve the simulation efficiency of financial derivatives pricing. In addition, the importance sampling method is used to optimize the selection, thereby making it closer to the theoretical values. The proposed method is easy to implement and has higher computational efficiency, which can ensure the financial benefits of users holding financial derivatives during the holding period. It can be seen that the Monte Carlo model-based variance reduction technology has high application value in the pricing of financial derivatives, and it is of great significance for the pricing of other products.

## 1. Introduction

With the continuous development of the world economy, financial derivatives become increasingly various. The financial derivatives are derived from basic financial instruments, such as currency, interest rate stocks, and commodities. Financial derivatives cannot exist independently, and their values largely depend on basic financial instruments. The global financial crisis triggered by the US subprime mortgage crisis in 2008 caused a huge blow to the major economic entities worldwide, making the world economy be into a recession. The financial markets of many developed countries also suffered heavy losses during the financial crisis. However, the most serious losses were the outbreak of the financial crisis and the United States, the most developed financial derivatives market. After research, the most important factors causing the crisis is considered to be the globalization of financial derivatives and the global proliferation of financial derivatives caused by lack of regulation. At present, there are more companies and users interested in financial derivatives. However, considering the value and risk of these products, there will be more considerations for the holding period of these derivatives [1].

RETRACTED

The Monte Carlo method has a wide range of applications in financial engineering. It can measure the number of occurrences of events and thereby the probability of occurrence of events. According to the law of large numbers and the central limit theorem in probability theory, the large number theorem can ensure that the estimated value obtained by the Monte Carlo method can gradually converge to the actual value according to the increase of the number of simulations, and the central limit theorem can give the error estimation range of the Monte Carlo model [2]. At the same time, since the Monte Carlo model is very adaptable, the conditional constraints are small when solving the problems. Financial products are usually priced to maximize the attractiveness of new and existing customers and to obtain the most theoretically priced prices; however, such pricing usually takes into account market share, high returns, and reduced competitors [3]. These financial derivatives are the major businesses of the bank, and the method of pricing the bank products should be based on the cost of the product and be determined flexibly in combination with the states of supply and demand, as well as the degree to which the customer is willing to pay.

Previous research has focused on the prediction of derivatives prices in various industries, while Monte Carlo models and variance reduction techniques can better predict the value of derivatives, which is vital for better judging the holding time. Therefore, considering the application of the Monte Carlo model in financial pricing and the related situation of financial derivatives pricing, the Monte Carlo model-based variance reduction technology is proposed to analyze the pricing problem of financial derivatives, which has a certain significance for the holding situations of users. It is expected that through the application of the Monte Carlo model, price fluctuations can be analyzed in the financial market to find the optimal holding time for users of financial derivatives, thereby reducing the risk of holding financial derivatives.

## 2. Literature review

With the collapse of the global fixed exchange rate regime and the continuous innovation in the financial sector, in addition to the traditional financial products, financial derivatives such as options, futures, and exchanges have developed rapidly. Monte Carlo is a commonly used statistical analysis method that can obtain an approximate solution to a problem based on economic indicators.

RETRACTED

### 2.1. Pricing of financial derivatives

Wang Yulin (2017) combed and summarized the relevant pricing methods of real estate derivatives to further understand the research process and achievements of real estate derivatives, thereby providing ideas for the subsequent research [4]. Rigatos and Zervos (2017) used stochastic differential equations and diffusion-type partial differential equations to describe financial derivatives and options, pricing models. Based on the descriptions, a method based on decomposing nonlinear partial differential equations that were grouped into a set of ordinary differential equations with respect to time was proposed. The accuracy of the model was verified by state estimation. The results showed that when the Black-Scholes PDE model was verified, the parameters in the Black-Scholes PDE model were inconsistent [5]. Hefter and Jentzen (2019) used the Cox-Ingersoll-Ross (CIR) process extensively in the latest financial derivatives pricing model and analyzed the convergence speed of the discretization method. The results showed that the discrete method can achieve up to one strong convergence order [6]. Jang and Lee (2019) proposed a Bayesian learning model in which the knowledge of the risk-neutral pricing structure was integrated, which provided a fairer price for the deep ITM and deep OTM options of few transactions. The research results showed that the established estimation model was compared with the machine learning option model. The machine learning prediction model had better prediction ability and showed better overall prediction performance [7].

### 2.2. Monte Carlo model

Spurzem and Giersz (2018) introduced a new method to analyze the gas models with different standards and performed dynamic analysis by Monte Carlo technology. The results showed that the standard theoretical model and the direct N-body model simulation results were more consistent, which also indicated that the method was an efficient and realistic model [8]. Wang et al. (2017) used the Monte Carlo model to analyze the impact of classification accuracy index and the variant on sample size, number of latent categories, category distance, and number of indicators, and their combinations on latent profile analysis. The results showed that there was a high correlation between Entropy value and classification accuracy, but it also changed with the sample size and index number. When other conditions were unchanged, the larger the sample size was, the smaller the Entropy value was, and the worse the accuracy of the classification was. If the sample size was small, the more the number of indicators was, the Entropy value also showed a better effect [9]. Zhang (2017) considered the real strategy of options trading and analyzed the trend of option value. In the process of using Monte Carlo in simulation, the value trend was analyzed from the perspective of intrinsic value, time value, and external volatility. The results showed that there was a certain correlation between the intrinsic value of the option and the time value. In addition, as the option time was shortened, especially on the option expiration date, the intrinsic value and time value of the option would decrease, while the external fluctuation rate and leverage would increase. Therefore, users who held the options were reminded to hold the options as early as possible before the expiration date [10].

RETRACTED

### 2.3. Variance reduction technology

Zhu and Chen (2018) used the Monte Carlo method to estimate the option price error and convergence rate. In addition, they utilized the least-squares method, the storage reduction technique, and the variance reduction technique to price the options of derivative securities. The research results showed that the standard deviation reduction effects of the control variable method and the dual variable method were obvious, and the dual variable method had a relatively average performance under different parameters. In addition, the effect of the control variable method depended on the correlation coefficient between the target assets, which was determined by the selected control variable. The convergence of the Monte Carlo method was improved by using a deterministic low-deviation sequence instead of a random point sequence [11]. Gao and Chen (2017) pointed out that under the Vasicek interest rate model, the pricing equations of ordinary bonds and European call options were deduced, and the discrete barrier options were priced based on them while the variances such as conditional expectation and importance sampling were used to reduce the variance and optimize the experimental analysis. The results showed that the Monte Carlo simulation method of conditional expectation and importance sampling and the two-variance reduction technology could be used to analyze the price of discrete obstacles, which could obtain more stable price data [12].

In summary, previous studies have focused on the prediction of derivatives prices in various industries, while the Monte Carlo model and variance reduction technology can better predict the value of derivatives. Therefore, in this paper, based on the Monte Carlo model of variance reduction technology, the value of financial derivatives pricing can make a good judgment on the holding time of financial derivatives holders, which is very important to judge the better time of holding.

RETRACTED

## 3. Methods

### 3.1. Monte Carlo method

The Monte Carlo method, also known as statistical simulation and random sampling, is a stochastic simulation method based on probability and statistical theory, which uses a random number (or more common pseudo-random number) to solve a variety of computational problems. Whether it is used on the computer is taken as an important sign. Therefore, although it belongs to the calculation method, it is quite different from the general calculation method. It links the solved problem to a fixed probability model and uses a computer to implement random sampling or statistical simulation, thereby obtaining an approximate solution to the problem [13].

With the continuous development of computer technology, the application of the Monte Carlo method becomes increasingly extensive. In addition, because of the excellent adaptability of the method, the calculation of integral, the solution of equations, and the calculation of eigenvalues can be easily obtained. Currently, the Monte Carlo method is mainly used to solve two types of problems, i.e., the randomness and certainty. Among these problems, the deterministic problem needs to establish a probability model. In such a process, the model is randomly observed, and its arithmetic mean is used to solve the approximate estimate of the model [14]. The random problem is that it is affected by random factors and needs to be solved by random sampling. The Monte Carlo algorithm is mainly used to study the probability density function, random number generator, sampling rule, simulation result record, error estimation, variance reduction technology, and parallel and vectorization [15–16]. The probability density function mainly generates a set of probability density functions describing a problem or system. Then, it generates a uniformly distributed random number of [0, 1] through a random number generator and randomly extracts obedience from these random numbers. For a given random variable, the corresponding simulation results are recorded, the errors of these results are estimated, and the variance reduction technology is used to reduce the number of calculations in the simulation process. Eventually, the method is operated [17–19].

When analyzing its convergence and error estimation, it is necessary to analyze its arithmetic mean value and expected value. The number of samples is denoted as N, the arithmetic mean of the samples is assumed as X_1_, X_2_, X_3_, … X_N_, as shown in Eq (1):

$${\bar{X}}_{N}=\frac{1}{N}\sum_{i=1}^{N}X_{i}$$ (1)

As an approximation of the solution, the sequence of variables in the sample is independent and identically distributed, and the probability value [20] can be obtained according to its expected value, as shown in Eq (2):

$$P\{\underset{N\to \infty }{\lim}{\bar{X}}_{N}-E\left(X\right)\}=1$$ (2)

However, since there is a certain error between the Monte Carlo approximation and actual value, and its variance value is shown in Eq (3):

$$0<\sigma^{2}=\int {\left(x-E\left(X\right)\right)}^{2}f\left(x\right)dx<\infty$$ (3)

In the above equation, f(x) is the distribution density function of X, then:

$$\underset{N\to \infty }{\lim}P\left(\frac{\sqrt{N}}{\sigma }\left|{\bar{X}}_{N}-E\left(X\right)\right|<x\right)=\frac{1}{\sqrt{2\pi }}\int_{-x}^{x}e^{-\frac{t^{2}}{2}dt}$$ (4)

If N tends to infinity, Eq (4) can be approximated as Eq (5):

$$P\left(\left|{\bar{X}}_{N}-E\left(X\right)\right|<\frac{\lambda_{\alpha }\sigma }{\sqrt{N}}\right)\approx \frac{2}{\sqrt{2\pi }}\int_{0}^{\lambda_{\alpha }}e^{-\frac{t^{2}}{2}dt}=1-\alpha$$ (5)

Therefore, the error of the Monte Carlo method can be obtained as shown in Eq (6):

$$\varepsilon =\frac{\lambda_{\alpha }\sigma }{\sqrt{N}}$$ (6))

In the above equation, *σ* indicates the fluctuation rate of the market, N indicates the times of simulation, *α* is the confidence degree, 1−*α* indicates the confidence level, the order of the error convergence speed is O(N^-1/2^), and the corresponding estimated value is as shown in Eq (7):

$$\hat{\sigma }=\sqrt{\frac{1}{N}\sum_{i=1}^{N}X_{i}^{2}-{\left(\frac{1}{N}\sum_{i=1}^{N}X_{i}\right)}^{2}}$$ (7)

As shown in Eq (6), the convergence speed is not related to the dimension of the problem sought, and its multiple integrals are proportional to the power of the dimension.

RETRACTED

### 3.2. Variance reduction technology-importance sampling

There are many methods for variance reduction. At present, the more common methods are controlled variable method, dual variable method, conditional expectation method, stratified sampling method, importance sampling method, related sampling method, and mixed-method [21].

Importance sampling increases the sampling probability of a given sample space and increases the sampling weights of important regions so that the events that have an important effect on the simulation results are more likely to occur, thereby reducing the variance and improving the sampling efficiency and estimation accuracy [22]. The importance of the original weight sampling principles is to select a density function g (x) and make it close to the shape of f (x). Herein, the density function g (x) is the envelope function [23]. Then, the expectation can be expressed by Eq (8):

$$\theta =E\left[h\left(X\right)\right]=\int h\left(x\right)f\left(x\right)dx=\int h\left(x\right)\frac{f\left(x\right)}{g\left(x\right)}dx$$ (8)

Sample estimation is performed on the data in g(x), and Eq (9) is obtained:

$$\hat{\theta }=\frac{1}{N}\sum_{i=1}^{N}h\left(X_{i}\right)w\left(X_{i}\right)$$ (9)

In the above equation, *w*(*X*_*i*_) is the original weight, i.e., f(x)/g(x).

RETRACTED

The standard weight can be expressed by Eq (10):

$$w^{*}\left(X_{i}\right)=\frac{w\left(X_{i}\right)}{\sum_{i=1}^{N}w\left(X_{i}\right)}$$ (10)

Thus, the corresponding standard expected value is obtained, as shown in Eq (11):

$$\theta =E\left[h\left(X\right)\right]=\frac{\int h\left(x\right)f\left(x\right)dx}{\int f\left(x\right)dx}=\frac{\int h\left(x\right)\frac{f\left(x\right)}{g\left(x\right)}g\left(x\right)dx}{\int \frac{f\left(x\right)}{g\left(x\right)}g\left(x\right)dx}$$ (11)

The operation of the estimation of g(x) is repeated. After repeating m times, the sample variance becomes Eq (12):

$$\theta^{'}=\frac{1}{m}\sum_{i=1}^{m}{\left({\hat{\theta }}_{i}-{\bar{\hat{\theta }}}_{i}\right)}^{2}$$ (12)

### 3.3. Asian option pricing

The risk-return characteristics of financial derivatives are different from those of general financial products. For example, an option can not only restrict market risk but also have a reservation effect on the market to retain profitable space. It is another characteristic that is different from the risk-return of basic assets. It is precise because of these advantages of financial derivatives that financial derivatives have won the favor of many investment enthusiasts, which makes financial derivatives gradually become an integral part of the basic asset portfolio.

As a financial derivative, options have a certain effect on risk avoidance and can avoid undesired consequences. In addition, it can largely benefit from good results. Currently, options have become one of the most versatile investments in financial instruments. In stock investment, continuous compounding is usually adopted. Also, the rise and fall of stock prices are generally irregular and will be affected by many factors. However, the randomness of the stock price also allows users to treat it as the value of a variable during the research process, which varies in an uncertain way over time. When the future prediction value of the variable in the stochastic process is only related to the current value of the variable and is independent of the past value, the stochastic process can be called as the Wiener process. The standard basic Wiener process is shown in Fig 1.

**Fig 1:** Basic Wiener process.

As shown in Fig 1, the behavior of the variable Z can be seen by the basic Wiener process generated by R, thereby predicting that the short time interval is a change of the variable Z. Asian options, also known as average price options, are derivatives of stock options and are based on lessons learned from the implementation of options, such as real options, virtual options, and stock options. Asian options are one of the most actively traded options in the current financial derivatives market. The difference between stock options and stock options in the usual sense is the limit on the execution price, which is the average price of the stock price for a period of time before the execution date. The difference from the standard option is that when the options income is determined on the maturity date, instead of using the market price of the underlying asset at the time, the average value of the asset price marked for a certain period of the contract period is used. Such a period is called the average period. When averaging the prices, the arithmetic mean or geometric mean is used.

RETRACTED

Assuming that an Asian option is priced at K and the expiration time is T, *P* represents the fee payable when purchasing an option, and its calculation can be expressed as Eq (13):

$$P={\left[\exp\left(\frac{1}{T}\int_{0}^{T}\ln\left(S_{t}\right)dt\right)-K\right]}^{+}$$ (13)

In the above equation, S_t_ represents the stock price at time t. However, since the currency is time-worthy, *P*' represents the current value of payment fees, and its calculation can be expressed as Eq (14):

$$P^{'}=\exp\left(-rT\right){\left[\exp\left(\frac{1}{T}\int_{0}^{T}\ln\left(S_{t}\right)dt\right)-K\right]}^{+}$$ (14)

Assuming that the option is bought at time t, P* represents the current value of payment fees, and its calculation can be expressed as Eq (15):

$$P^{*}=-f_{c}+\exp\left(-rT\right){\left[\exp\left(\frac{1}{T}\int_{0}^{T}\ln\left(S_{t}\right)dt\right)-K\right]}^{+}$$ (15)

The return of the lookback option has a certain relationship with the maximum value of the underlying asset before the maturity date. The simulation results are shown in Fig 2:

**Fig 2:** Simulation results of option pricing.

The pricing of fixed-looking call options and European call options is related to the strike price, while the price of the fixed-back call option is higher than the corresponding European call option. If the risk does not pose a threat, the expected yield of the stock is the risk-free rate. Therefore, the expected stock price on the maturity date will be higher than the average stock price during the effective period. At this time, the price of the floating look-up call option will be higher than the price of the corresponding Asian call option.

The value of the lookback option mainly depends on the highest or lowest price of the underlying asset that can be observed during the life of the option. In particular, there is an analytical solution to the pricing of the option under the continuous model, i.e., the lowest price or the highest price of the stock can be obtained when the continuous observation is performed. However, since the price of the underlying asset is discrete, the price under the continuous model can only be considered as an approximation of the actual price. As the frequency of observation increases, the probability of observing the extreme value increases. At this time, the price of the lookback option also shows an upward trend with the increase of the observation frequency. The Monte Carlo simulation of the European option is shown in Fig 3:

**Fig 3:** Monte Carlo simulation flow of European options.

RETRACTED

The Asian option differs from the standard option. In such a case, when the options income is determined on the maturity date, the average value of the asset price of a short time target within the short time of the option is used to determine the price average operation. The method is mainly to avoid malicious manipulation of stock prices, and it can also reduce the insider trading of internal employees and damage the interests of the company to a certain extent.

## 4. Results and discussions

It is supposed that the current price of a stock is 50, the market volatility is *σ*, which is set at 40%, the risk-free rate is 10%, and the expiration is 3 months. According to the European lookback option, the value of the call option is 8.03. The Monte Carlo model-based variance reduction technology is used to calculate the price of the option, and the possible risks in the 3 months are also compared to simulate the stock path, thereby setting the price observation point and finding the lowest stock price as the exercise price. Then, the profit and loss of the option are calculated. The trends of log prices of ten-year Treasury bill futures and spots in 2015–2017 are collected, and the data in Fig 4 are obtained:

**Fig 4:** Trends of log prices of ten-year Treasury bill futures and spots in 2015–2017.

As shown in Fig 4, the price has decreased in recent years, and it is necessary to predict future trends.

Therefore, the data are assumed to be solved in Excel VBA, and the results of Table 1 are obtained:

**Table 1:** Simulation results.

Number of simulations	Equity value when the price observation point is 100 times	The value of the option when the price observation point is 1000 times	Number of simulations	Equity value when the price observation point is 100 times	The value of the option when the price observation point is 1000 times
1000	7.4724	7.6051	6000	7.5791	7.9262
2000	7.5616	7.7757	7000	7.5204	7.9254
3000	7.3442	7.7219	8000	7.6163	7.8825
4000	7.4721	7.7763	9000	7.6014	7.9051
5000	7.4746	7.7768	10000	7.4794	7.8861

In the hypothesis that the stock price obeys several Brownian movements, the stock price movement path can be further stimulated. When the static comparison is made, the time value of the currency is not considered, and the calculated theoretical value and the option value are increased in the simulation process. The error will become increasingly smaller. When performing dynamic comparison, according to the big number theorem, if the number of simulations increases, the simulated value will be closer to the true value. According to the central limit theorem, the deviation in the simulation process will also be concentrated in a certain range.

RETRACTED

It requires to transform the number of simulations while controlling other conditions. From the results, the relative error between the analog and real values is simulated. Afterward, it is necessary to use the Monte Carlo model-based variance reduction technology to carry out simulation experiments to ensure that the dimension is floating in a small range, which can avoid the adverse effects of random scatter on the experimental results.

By analyzing the simulation data results, the average absolute error data of different simulation times under important sampling is obtained, as shown in Fig 5:

**Fig 5:** Average absolute error of different simulation times under importance sampling.

In addition, according to the above simulation calculation results, the convergence of Fig 6 is obtained:

**Fig 6:** Convergence process of the option value.

As shown in Fig 6, during the continuous observation, the price change is small, and the lowest price and the highest price of the option can be accurately understood.

In summary, based on the importance sampling method in the variance reduction technology, the Monte Carlo model is used to simulate the hypothesis data. It can be seen that as the observations increase, the prediction results are better. In addition, with the increase with frequency, i.e., the observation time is shortened, the possibility of observing the highest price and the lowest price is greater. Since it can solve this problem well when the input is significantly uncertain during the simulation, the Monte Carlo model has been accepted and adopted by many scholars. The Monte Carlo model is performed under certain assumptions, which is different from the real trading environment and has a certain impact on the empirical results. The accuracy of the Monte Carlo's calculation results is high. When a certain number of simulations are reached, the accuracy of the results is extremely high. The disadvantage of the Monte Carlo method is that the computational workload is huge, and it takes more time. However, technology is constantly improving, and the performance of all aspects of computers has been greatly improved. The computing efficiency of the Monte Carlo model has been correspondingly improved.

RETRACTED

## 5. Conclusions

Based on the variance reduction technology, the Monte Carlo model that can effectively analyze the financial price is added. Through the simulation of the test and the analysis of the value of the stock price at 100 and 1000, the estimated value is reduced. The actual value error helps investment enthusiasts find the best holding time for financial derivatives holdings, as well as reducing the holding risks. The application of variance reduction based on the Monte Carlo model in the pricing process of financial derivatives has a certain guiding role in the pricing of financial derivatives, which can help related companies adopt better strategies in pricing and attract customers while expanding the market share. In addition, at the same time, the market risk can be adjusted to varying degrees to avoid bringing greater losses to financial derivatives, thereby providing certain ideas for investment enthusiasts in selecting financial derivatives. This study has preliminarily researched and applied the Monte Carlo model; however, it lacks comparative analysis with other prediction models to find the shortcomings of the Monte Carlo model in data prediction. In the subsequent study, other commonly used price analysis models will be analyzed to find out how to minimize the error between the simulated value and the actual value, thereby reducing the transaction costs, accelerating the transaction speed, and increasing the returns on investment.

## Supporting information

S1 Data (DOCX)
